The article "Transmission and Drug Resistance Characteristics of Human Immunodeficiency Virus-1 Strain Using Medical Information Data Retrieval System" was published in 2022. Journal: Comput Math Methods Med.

# Transmission and Drug Resistance Characteristics of Human Immunodeficiency Virus-1 Strain Using Medical Information Data Retrieval System

**DOI:** 10.1155/2022/2173339

**Published:** 2022-06-13

**Authors:** Ning Wang, Hui Qi, Yong Deng, Weiwei Yu, Zhong Chen

**Affiliations:** ^1^Department of Infection and Immunology, The First Hospital of Changsha City, Changsha, 410000 Hunan, China; ^2^Postgraduate School, Changsha Hospital Affiliated to Nanhua University, Changsha, 410000 Hunan, China

## Abstract

This study was aimed at exploring the transmission and drug resistance characteristics of acquired immunodeficiency syndrome (AIDS) caused by human immunodeficiency virus-1 (HIV-1). The query expansion algorithm based on Candecomp Parafac (CP) decomposition was adopted to construct a data information retrieval system for semantic web and tensor decomposition. In the latent variable model based on tensor decomposition, the three elements in the triples generated feature vectors to calculate the training samples. The HIV patient data set was selected to evaluate the performance of the system, and then, the HIV gene resistance of 213 patients was retrospectively analyzed based on the electronic medical records. 43 cases showed failure of ribonucleic acid drug resistance, the ART virological failure rate was 24.43% (43/213), and one case was not reported. There was 1 case of RNA hemolysis that could not be detected. There were 50 resistant cases of nonnucleotide reverse transcriptase inhibitors (NNRTI), accounting for 29.94% (50/167), and there were 17 resistant cases of nucleotide reverse transcriptase inhibitors (NRTI), accounting for 10.18% (17/167) of all mutation cases. Among the HIV-1 strains, 19 cases failed the detection of drug resistance sites in the integrase region, and mutations in the integrase region were significantly more than those in the protease region. There were 12 types of HIV-1 strains with drug-resistant mutations. The fusion technical scheme constructed in this study showed excellent performance in medical information retrieval. In this study, the characteristics of HIV-1 of AIDS patients were analyzed from different directions, and effective treatment was performed for patients, so as to provide reference for clinical diagnosis of AIDS patients.

## 1. Introduction

Acquired immune deficiency syndrome (AIDS) refers to that human immunodeficiency virus (HIV) which invades the human immune system, causing immune function damage and various opportunistic infections in the body [1–4]. At this stage, there is no specific treatment method for AIDS [5–8]. Virus strains may have drug resistance mutations due to natural mutations or the selection of antiviral drugs. After mutations, more adaptable strains become dominant strains and spread further [9–11]. HIV includes two types, HIV-1 and HIV-2. HIV-1 is the main strain circulating globally in the new stage. The M, N, P, and O of HIV-1 and HIV-2 are relatively weak in pathogenicity, mainly in Central Africa and West Africa, while European and American countries are dominated by type B strains [12, 13]. At present, HIV-1 drug resistance data and drug resistance mechanisms are mainly derived from B subtype, but B subtype infection only accounts for 10% of the global HIU-1 infection population. Subtype C is the most prevalent HIV-1 subtype in the world. Due to differences in intrinsic adaptability and replication ability, the accumulation of drug-resistant mutations in different subtypes of infected individuals may be different, and drug selection pressure has different effects on drug-resistant mutations in different subtypes of strains. New drug resistance mutations are being reported, and some unexplained drug sensitivities may explain the results of genotypic resistance [14–16]. Research on drug resistance of the main HIV-1 subtypes prevalent in my country and summarizing the characteristics of drug resistance of patients with failed antiviral treatments is very important for clinical treatment [17].

The article "Transmission and Drug Resistance Characteristics of Human Immunodeficiency Virus-1 Strain Using Medical Information Data Retrieval System" was published in 2022. Journal: Comput Math Methods Med.

The continuous development of information and the diversified information demands have accelerated the process of big data [18]. Extended search is to screen the currently available information resources and adjust the scope of the search based on the reduced content. The formulation of the search scope needs to be divided into more levels and steps according to the needs [19–21]. At this stage, the molecular epidemiological investigation of HIV-1 is not clear, so it is necessary to conduct retrospective research on the genotypic characteristics of HIV-1 and the emergence of drug resistance characteristics.

Based on electronic medical records and oriented to medical literature retrieval for diagnosis and treatment decision support systems, an enhanced medical information retrieval system was constructed in this study. It integrated structured and unstructured data sources, combined the supervised learning methods for automatic query expansion to improve the effect of information retrieval, and analyzed the drug resistance characteristics of HIV-1 strains of AIDS patients from different directions. This study is aimed at providing a reference for clinical diagnosis of AIDS patients.

## 2. Materials and Methods

### 2.1. Research Objects

This study retrospectively analyzed 213 patients who were treated in hospital. The data were mainly sourced from the *Archives of Antiretroviral Treatment for AIDS Patients* collected by the Municipal Center for Disease Control and Prevention and the *National Handbook of Free AIDS Antiretroviral Treatment* collected by the state. The diagnostic criteria and the diagnostic criteria stipulated in the *Guidelines for the Diagnosis and Treatment of AIDS* in China jointly promulgated by the Chinese Medical Association and the Ministry of Health in 2004. The antiretroviral failure standard referred to the *National Handbook of Free AIDS Antiviral Drug Treatment*. The prescribed standards were divided into virological failure, immunological failure, and clinical failure.

The article "Transmission and Drug Resistance Characteristics of Human Immunodeficiency Virus-1 Strain Using Medical Information Data Retrieval System" was published in 2022. Journal: Comput Math Methods Med.

### 2.2. HIV-1 Introduction

HIV-1 viral load was based on the *Guidelines for HIV-1 Viral Load Determination and Treatment Assurance (2013 Edition)*. The EasyQ viral load meter (France, BioMérieux) was adopted to test the HIV viral load in plasma. 100 copies/mL was defined as the lowest detection limit, and the operation process was carried out strictly in accordance with the instructions. Then, the self-built genotype drug resistance test method was adopted to extract the viral ribonucleic acid (RNA) from the plasma using the QIAamp Viral RNA Isolation Kit according to the *HIV-1 Genotype Drug Resistance Test and Quality Assurance Guidelines (2013 Edition)*. Nested polymerase chain reaction (PCR) was adopted for two rounds of amplification, covering the entire gene sequence and the reverse transcriptase codon sequence. Taking the extracted RNA was the template, and the gene sequence amplification was performed using reverse transcription PCR (RT-PCR) and nest-PCR methods. The genotype was determined based on the National Center of Biotechnology Information (NCBI) genotyping tool. The calibrated sequence was submitted to the HIV drug resistance database of Stanford University (http://hivdb.Stanford.edu) for online analysis of HIV drug resistance-related mutations and drug resistance. The degree of drug resistance was judged according to Table 1.

### 2.3. Data Mining

The development and application of medical information technology have produced a huge amount of data, so it is necessary to dig out potentially useful information from a large amount of obscure data and observe and analyze more useful knowledge from different angles. Data mining technology uses computer science, statistics, artificial intelligence, and other technologies to intelligently and efficiently analyze the objects in the target database and intelligently summarize or predict potential models to make reasonable decisions for the individual. The basic process of data mining mainly includes target understanding, data collection, data preprocessing, model building, model evaluation, and implementation. It can be regarded as a cyclical operation process. If the target set during the excavation is not reached, it should return to the previous one without making adjustments and then perform the operation.  Figure 1 shows the flow chart of data mining.

The article "Transmission and Drug Resistance Characteristics of Human Immunodeficiency Virus-1 Strain Using Medical Information Data Retrieval System" was published in 2022. Journal: Comput Math Methods Med.

It was supposed that in the database *W* = {*P*1, *P*2, ⋯*Pn*}, *Tx* = {*L*1, *L*2, ⋯..*Ln*}, *n* represented the number of items, *Tx* was a transaction, *Km* (*m* = 1, 2, 3, ⋯, *n*) was the data item (Item), and the value in the data table was the item. The set *F* = {*f*1, *f*2, *f*3 ⋯ *fn*} in the *W* database was selected, and *Q* was to represent any subset. Each field in the data table was close to the item in the set, the length of *Q* was set to *y*, *Q* can be called *y*-itemset, for example, set *I* = {product *A*}, *F* was *f*-itemset.

If set *f* ∈ *F*, the frequency of *f* appearing in *F* was *U*, and the total length of set *f* was *M*; then the support of *f* was expressed as follows:

(1) $$\begin{array}{c} \text{Support}\left(F\right)=\frac{xn}{N}=\frac{U}{y}. \end{array}$$

Support*T* described the proportion of itemsets relative to itemsets, *n* was the number of occurrences, and *N* was the total number of things.

In a transaction, 1-itemset *H* = {item *H*}, *S* = {item *S*} has *H*⟶*S*. If *H* was selected, *S* must also be selected. The support of (*H*⇒*S*) represented the frequency of *HS* cooccurrence; the equation was as follows:

(2) $$\begin{array}{c} \text{Support}\left(H\Rightarrow S\right)=\text{Support}\left(H\cup S\right)\frac{\left(H\cup S\right)}{\left|F\right|}\times 100\%. \end{array}$$

The association rule (*H*⇒*S*) was found, *H* ∈ *F*, *S* ∈ *F*, and *H*∩*S* = *Φ*; then, the confidence of the data set was expressed as follows:

(3) $$\begin{array}{c} \text{Confidence}\left(H\Rightarrow S\right)=P\left(Y\left|X\right.\right)\frac{P\left(XY\right)}{P\left(X\right)}\times 100\%=\frac{\text{Sup}\left(XY\right)}{\text{Sup}\left(X\right)}\times 100\%. \end{array}$$

In the set *F*, the confidence of the rule *R* was expressed as the probability that *Y* would also appear under the condition that *X* appears, so as to show the reliability of this rule.

Minimum support shows the minimum threshold that valuable knowledge must meet, which shows the lowest importance of discovering this rule. Only when the minimum support degree is satisfied can it show its practical significance.

The minimum level of reliability that valuable knowledge must meet is the minimum confidence level (Minimum Confidence). Compared with the support degree, the confidence degree is used to measure the credibility of the excavated association rules; that is, the higher the confidence degree, the higher the credibility degree. Low credibility will be discarded.

The article "Transmission and Drug Resistance Characteristics of Human Immunodeficiency Virus-1 Strain Using Medical Information Data Retrieval System" was published in 2022. Journal: Comput Math Methods Med.

### 2.4. Medical Information Retrieval System

The method and technology of obtaining medical information through a new type of retrieval is called information retrieval. In this study, the medical information retrieval system is constructed by enhancing semantics, comprehensively supervised learning, and automatic query expansion to improve the information retrieval effect. The first is to input the query expansion words and then select the documents. The semantic expansion model selected based on tensor decomposition was adopted to expand the query words, search and sort the obtained files, and then obtain the search results. Query expansion includes two parts of sources: one is structured data, and the other is unstructured data. The combination of the two types of data can achieve better results in information retrieval.  Figure 2 shows the framework of semantic-enhanced information retrieval system.

### 2.5. Three-Dimensional Tensor Representation

In actual information retrieval tasks, large-scale data document collections and limited labeled samples cannot support triple query expansion. The semantic web triples are adopted to assist query and document relevance to help retrieve relevant literature on treatment. In the data knowledge base, there are problems of incompleteness, sparsity, and noise, and tensors are used to represent triples. Each associated triple represents the value in the tensor and plays an important role in the analysis process. The specific schematic diagram is illustrated in Figure 3.

### 2.6. The Query Expansion Algorithm Based on Candecomp Parafac (CP) Decomposition

Tensor representation can provide good prediction performance under the condition of coefficients. Compared with traditional methods, it can significantly emphasize the impact of different semantic relationships on correlation analysis. In the process of analyzing the relevance of different semantic triples, if *R*_*i*_ is used to represent the query word category, *Q*_*k*_ is used to represent the semantic relationship, and *A*_*k*_ is used to represent the document word type; the corresponding feature vectors are generated after decomposition. According to the inner product of feature vectors, the triples are scored, and *M* is selected to represent it. The calculation equation was as follows:

(4) $$\begin{array}{c} f\left(R_{i},Q_{j},A_{k}\right)=\overset{M}{\underset{r=1}{\sum }}R_{ir}Q_{jr}A_{kr}. \end{array}$$

The initial value of the important score of the triple selected in the marked sample contains the value in the original quantity, and the calculation equation was as follows:

(5) $$\begin{array}{c} {\text{C}}_{\text{f}}\left(R_{i},Q_{j},A_{k}\right)=\frac{{\text{C}}_{\text{r}}\left(R_{i},Q_{j},A_{k}\right)}{{\text{C}}_{\text{f}}\left(R_{i},Q_{j},A_{k}\right)}. \end{array}$$

C_f_(*R*_*i*_, *Q*_*j*_, *A*_*k*_) represents the number of triples (*R*_*i*_, *Q*_*j*_, *A*_*k*_) in the marked sample, and C_r_(*R*_*i*_, *Q*_*j*_, *A*_*k*_) represents the number of triples (*R*_*i*_, *Q*_*j*_, *A*_*k*_) extracted from the marked relevant documents and query terms. Initial value ∈ (0, 1). The tensor CP decomposition used the alternating least squares algorithm to perform tensor decomposition calculation on the semantic relations in the prediction data set.

The article "Transmission and Drug Resistance Characteristics of Human Immunodeficiency Virus-1 Strain Using Medical Information Data Retrieval System" was published in 2022. Journal: Comput Math Methods Med.

The CP decomposition of a three-dimensional tensor can be represented by a factor matrix, as follows:

(6) $$\begin{array}{c} Y\approx Y^{\prime }=\left[A,B,C\right]. \end{array}$$

The expanded matrix form was expressed as follows:

(7) $$\begin{array}{c} Y\approx Y^{\prime }\left(1\right)={\left({\left(C⊙B\right)}^{N}\right)}^{+}. \end{array}$$

⊙ represents the Khatri-Rao product, and ^+^ represents the Moore-Penrose pseudoinverse, and the matrix *A* could be expressed as

(8) $$\begin{array}{c} A=Y\prime_{\left(1\right)}={\left({\left(C⊙B\right)}^{N}\right)}^{+}. \end{array}$$

Then, the Khatri-Rao product attribute was expressed as

(9) $$\begin{array}{c} {\left(C⊙B\right)}^{N}\left(C⊙B\right)=C^{N}C*B^{N}\left.B\right). \end{array}$$

The below equations were found.

(10) $$\begin{array}{c} W^{+}=W^{\text{N}}W^{+}W^{N},\\ {\left({\left(C⊙B\right)}^{N}\right)}^{+}=\left(C⊙B\right){\left(\left(C^{N}C\right)*\left(B^{N}B\right)\right)}^{+}. \end{array}$$

Then, equation (9) can be obtained as follows:

(11) $$\begin{array}{c} A=Y\prime_{\left(1\right)}\left(C⊙B\right){\left(\left(C^{N}C\right)*\left(B^{N}B\right)\right)}^{+} \end{array}$$

Equation (11) can perform iterative and alternate calculations for tensor decomposition. For labeled samples, using tensor decomposition to evaluate semantics was very important. The equation for constructing tensors is shown in

(12) $$\begin{array}{c} Y^{\prime }=Y*U+Y*\left(1-U\right). \end{array}$$

In the equation above, *U* represents the observed element of marked *Y*, *Y* represents the tensor filled with missing values, and 1 represents the tensor of element 1. In the calculation process, only the observed values were considered. The optimized function was expressed as

(13) $$\begin{array}{c} f_{u}\left(A,B,C\right)=\overset{j}{\underset{i=1}{\sum }}\overset{j}{\underset{j=1}{\sum }}\overset{k}{\underset{k=1}{\sum }}{\left(U_{Yijk}\left(Y_{ijk}-Y\prime_{ijk}\right)\right)}^{2}, \end{array}$$

(14) $$\begin{array}{c} U_{Yijk}=\left\{\begin{array}{c} 1,\;\text{if }Y_{ijk}\text{ know},\\ 0,\;\text{if }Y_{ijk}\;\text{is }missing\;value. \end{array}\right. \end{array}$$

In practical applications, the selection of rank was close to the original tensor. The larger the rank, the smaller the error. Therefore, the known elements can be used to calculate the fitting situation and gradually increase the rank value and finally decompose the parameters. In the proposed system, for the semantic expansion mode, calculation was not allowed in the process of specific query, so it would not affect the efficiency of the system.

The article "Transmission and Drug Resistance Characteristics of Human Immunodeficiency Virus-1 Strain Using Medical Information Data Retrieval System" was published in 2022. Journal: Comput Math Methods Med.

### 2.7. CP-ALS Decomposition Algorithm of 3D Tensor

The complexity of tensor calculation was constantly increasing, which was also one of the shortcomings of calculation. In the proposed system, tensor decomposition was used to evaluate the mode of semantic expansion, which was not necessary to be calculated in the process of requiring specific queries, so that it would not affect efficiency of the system.

Figure 4 illustrates the process of the ALS algorithm. The *r* in the figure represents the number of iterations. In the latent variable model based on tensor decomposition, the three elements in the triples generated feature vectors to calculate the training samples.

### 2.8. Data Set

In order to evaluate the performance of the constructed information retrieval system, the HIV patient data set was used, which was oriented to the diagnosis and treatment decision support system. The medical literature was retrieved based on query statements generated by electronic medical records. The data set provided query statements, document collections, and evaluation samples. Summary represents a simplified summary of report information, type represents the type of information required, and description represents a complete report. PudMed Central (PMC) is a literature database that provides free full text for the fields of biomedicine and life sciences. The task of the data set is to retrieve relevant documents from the document collection based on the query and to support the diagnosis or treatment plan of the corresponding case.

### 2.9. Statistical Methods

The survey data processing in this study was analyzed by SPSS19.0 version statistical software. The measurement data conforming to the normal distribution were expressed by the mean ± standard deviation ($\bar{x}\pm s$), and the nonconforming count data was expressed by the frequency and frequency (%). The *t*-test data was adopted, and a chi-square test was performed for quality comparison. The difference was statistically significant at *P* < 0.05; otherwise, it was not significant.

The article "Transmission and Drug Resistance Characteristics of Human Immunodeficiency Virus-1 Strain Using Medical Information Data Retrieval System" was published in 2022. Journal: Comput Math Methods Med.

## 3. Results

### 3.1. Objects of Investigation

Using data mining in the established gene bank, 4,817 HIV patients included in this study were identified. The obtained Pol gene sequence infected 3,716 cases, the amplification rate was 77.14%, the average age was 39 years, and the transmission route was mainly heterosexual transmission, accounting for 73.09% (Table 2).

### 3.2. Evaluation of the System

For large-scale document collections, it is difficult to implement complete relevance annotation. For the incomplete test set, the evaluation parameters choose inferred average precision (infap), inferred normalized discounted Cumulative gain (infndgg), and precision at rank10 (p10). The incremental PRF system and Solr are used as the baseline system to evaluate the performance of the medical information data retrieval system. The system can effectively improve the accuracy of retrieval and achieve consistent results in measurement parameters. The specific comparison on performance evaluation of medical information retrieval system is illustrated in Figure 5.

The support vector machine (SVM) was used to test the classification effect, and the radial basis function (RBF) and linear functions were used to evaluate the accuracy. The results are shown in Figure 6. It can be observed that the SVM of linear kernel function and the SVM of RBF were not very satisfactory and may be affected by many factors such as noise.

### 3.3. Comparison on Accuracy

The average accuracy of least squares decomposition machine (Fm-als) used in this study is shown in Figure 7. The average accuracy of Fm-als was 0.793, the average accuracy of svm-RBF was 0.546, and the average accuracy of svm-linear was 0.561. Therefore, the accuracy of Fm-als was significantly higher than that of other methods, and the difference was significant (*P* < 0.05).

### 3.4. Basic Situation of Research Objects

In the study, 43 cases of RNA drug resistance test failed, and the basic conditions of the patients who failed the test were statistically analyzed. The results are shown in Table 3. The ART virological failure rate was 24.43% (43/213). The results of gender showed that males were higher than females, and unmarried cases were higher than married or cohabiting cases and separated cases. The Han nationality showed significantly more cases than the minority nationalities.

### 3.5. Strain Mutation

A total of 213 strains were studied, 43 of which failed the RNA drug resistance test, and one test report did not come out. There was 1 case of RNA hemolysis that could not be detected. There was 1 DNA showing that the detection of DNA and RNA drug resistance sites failed.  Table 4 shows the mutations at the drug resistance site of the HIV-1 strain. There were 50 cases of drug resistance of nonnucleotide reverse transcriptase inhibitors (NNRTI), accounting for 29.94% (50/167).

The article "Transmission and Drug Resistance Characteristics of Human Immunodeficiency Virus-1 Strain Using Medical Information Data Retrieval System" was published in 2022. Journal: Comput Math Methods Med.

There were 17 cases of drug resistance of nucleotide reverse transcriptase inhibitors (NRTI), accounting for 10.18% (17/167) of all mutation cases. Each mutation site and mutation rate are shown in Table 5.

### 3.6. Mutant Strain Type in Drug Resistance

There were 12 types of virus strains with drug resistance mutations, as shown in Table 6. A total of 167 cases of drug resistance mutations occurred in this study. The number of cases with different virus strains is shown in Table 6.

### 3.7. Mutation Sites in the Protease Region and Integrase Region

Of the 213 cases in this study, 19 cases failed to detect the drug resistance site in the integrase region, and 1 case was retested on the drug resistance site in the integrase region. The mutation sites of the protease region and the integrase region are shown in Table 7. The mutations in the integrase region were significantly more than those in the protease region.

## 4. Discussion

Since the Chinese government issued the “Four-Free and One-Care” policy for AIDS prevention and treatment in 2003, free antiretroviral treatment for AIDS has been launched in China, providing free antiretroviral treatment for AIDS patients. HIV replicates, evolves, and spreads under the pressure of drugs. The selective pressure of drugs causes the virus to quickly produce drug resistance, which obviously changes the evolutionary characteristics of the virus in its natural state [22]. Among the free antiviral treatment formulas, there are 6 kinds of imitation antiviral drugs (didanosine (DDI), azidothymidine (AZT), 2′,3′-didehydro-3′-deoxythymidine (D4T), lamivudine (3TC), nevirapine (NVP), and efavirenz (EFV)) to compose 6 formulas such as AZT/DDI/NVP and AZT/3CT/NVP. Antiviral therapy can reduce the speed of virus replication for HIV patients and improve the body's immunity [23].

Clare et al. [24] showed that the incidence of drug resistance of HIV subtype B after antiviral treatment was 7.1%. Guan et al. [25] suggested that the mutation rate of subtype B and subtype C was 4.71% and 1.05%, respectively, and the prevalence of low-level monitored drug-resistant mutations was predicted to be 2.1%. There were 12 virus strains with subtype B-resistant mutations in this study, and the proportion of subtype B cases was 4.09% (7 out of 176), which was basically consistent with Guan's research results. The proportion of subtype C cases was 5.99% (1 in 176), which was higher than that of Guan's, which may be related to the region of the study population. In this study, 19 of the 213 cases failed to detect integrase region drug resistance sites, and 1 case was retested for integrase region drug resistance sites. There were more mutations in the integrase region than in the protease region. Different subtypes of HIV-1 strains have different drug-resistant mutation patterns compared with subtype B, possibly because subtype-specific genetic barriers can play a certain role in the occurrence of drug-resistant mutations. The emergence of drug resistance strains causes the virus to be insensitive to or less sensitive to drugs, which is the main reason for the failure of antiviral treatment [26]. Silva et al. [27] studied 75 patients who received antiretroviral therapy, of which 13 patients (17.3%) had a TDR (95% confidence interval: 9.6-27.8). Drug resistance mutations to NNRTI were dominant (14.7%), followed by NRTI (5.3%) and protease inhibitors (PI) (1.3%). In this study, there were 17 cases of drug resistance of nucleotide reverse transcriptase inhibitors, accounting for 10.18% (17/167) of all mutation cases. 43 cases failed the RNA drug resistance test, and one test report did not come out. There was 1 case of RNA hemolysis that could not be detected. There was 1 DNA showed that the detection of DNA and RNA drug resistance sites failed. There were 50 cases of drug resistance of NNRTI, accounting for 29.94% (50/167). Different epidemiological characteristics show diversification in the distribution of the number of HIV drug resistance cases in the population. Different genders, different marital status, and infection routes all show that the transmission routes of HIV drug resistance tend to be diversified. In this study, it was found that the mutation sites in NNRTI were significantly more than those in the NRTI region, and mutations also occurred in the integrase region and the protease region. There were 43 patients who failed in this study, which should also increase the management of drug resistance. The types of drug resistance and the degree of drug resistance of various drugs can be used as the basis for case adjustment and medication, which showed reference value and guiding significance for clinicians' medication.

The article "Transmission and Drug Resistance Characteristics of Human Immunodeficiency Virus-1 Strain Using Medical Information Data Retrieval System" was published in 2022. Journal: Comput Math Methods Med.

## 5. Conclusion

Based on electronic medical records and oriented to medical literature retrieval for diagnosis and treatment decision support systems, an enhanced medical information retrieval system was constructed in this study. It integrated structured and unstructured data sources, combined the supervised learning methods for automatic query expansion to improve the effect of information retrieval, and analyzed the drug resistance characteristics of HIV-1 strains of AIDS patients from different directions. The semantic web and tensor decomposition constructed in the study could perform effective data mining in the data retrieval system, and the fusion technical solution showed excellent performance in medical information retrieval. There were still some shortcomings in this study. The three-tuple relationship network was proposed in the article only. If the four-tuple relationship was constructed, whether semantic analysis and tensor decomposition were more accurate and effective required effective and in-depth discussion in the next step.

## Figures and Tables

**Figure 1:** Schematic diagram of data mining process.

**Figure 2:** Framework of semantic-enhanced information retrieval system.

**Figure 3:** Schematic diagram of tensor representation of triples.

**Figure 4:** Schematic diagram of the ALS algorithm process.

**Figure 5:** Comparison on performance evaluation of medical information retrieval system. ∗ indicates statistically significant difference, *P* < 0.05.

**Figure 6:** Classification accuracy evaluation of support vector machine.

**Figure 7:** The average accuracy of the classification method. ∗ indicates that the difference was significant (*P* < 0.05).

**Table 1:** Judging criteria for degree of drug resistance.

Degree of drug resistance	Score
Sensitive	0-9 points
Potential drug resistance	10-14 points or more
Low resistance	15-29 points or more
Moderately resistant	30-59 points or more
Highly resistant	60 points or more

**Table 2:** Basic information of infected persons.

Variable	Number of cases (cases)	Percentage (%)
Total	3716	
Gender		
Female	1349	36.30%
Male	2367	63.70%
Age		
16-25	511	13.75%
25-50	1876	50.48%
>50	1208	32.51%
Unknown	121	3.26%
Way for spreading		
Same-sex transmission	490	13.19%
Heterosexual transmission	2716	73.09%
Injecting drug use	198	5.33%
Others	312	8.40%

**Table 3:** Strains at NRTI drug resistance mutation sites.

Basic situation	6–12 (months)	13–24 (months)	25–36 (months)	≥37 (months)	Proportion (%)	*χ* ^2^	*P*
Gender							
Male	13	6	5	3	62.79	0.000	1.000
Female	4	0	2	10	37.21		
Marital status							
Married or living together	5	2	1	3	25.58	19.37	0.000
Divorced or separated	2	0	2	1	11.63		
Unmarried	15	1	3	8	62.79		
Nationality							
Han	12	8	5	3	65.12	2.189	0.123
Minorities	9	3	2	1	34.88		
Way for spreading							
Sexual transmission	21	6	3	1	72.09		
Others	5	2	4	1	27.91		

**Table 4:** Strain mutation site in NNRTI drug resistance.

Mutation site	Number of cases NNRTI	NNRTI mutation rate (%)
V106V1	4	8.0
V179E	16	32.0
V1061	5	10.0
V179VD	1	2.0
V179D	10	20.0
V197DN	1	2.0
V1791	1	2.0
K103N	9	18.0
V1081	1	2.0
V108V1	3	6.0
M2301	1	2.0
M230L	3	6.0
E138G	2	4.0
H221HY	1	2.0
Y188C	1	2.0
Y188L	2	4.0
Y181YC	1	2.0
Y181C	2	4.0
P225PH	1	2.0
V106M	2	4.0
K10P	1	2.0
G190A	3	6.0
G190S	3	6.0
K101E	1	2.0
E138EK	1	2.0
G140K	1	2.0
G163R	1	2.0
E138EG	1	2.0
K101KE	1	2.0
K103KNRS	1	2.0
V179T	1	2.0

The article "Transmission and Drug Resistance Characteristics of Human Immunodeficiency Virus-1 Strain Using Medical Information Data Retrieval System" was published in 2022. Journal: Comput Math Methods Med.

**Table 5:** Strain mutation site in NRTI drug resistance.

Mutation site	Number of cases	NRTI mutation rate (%)
M184MT	1	5.82
M184V	9	52.94
M184MIV	3	17.65
M1841	2	11.76
Y115F	1	5.82
K65R	2	11.76
L74L1	4	23.53
K70KT	1	5.82
K70Q	1	5.82
K70E	1	5.82
K219R	1	5.82
K219KE	1	5.82
D67N	1	5.82
T215TA	1	5.82
T69TADN	1	5.82
R70T	1	5.82
V179D	1	5.82

**Table 6:** Mutant strain type in drug resistance.

Virus strain	Number of cases (cases)	Proportion (%)
CRF01-AE	23	13.77
CRF55-01B	8	4.79
B	7	4.19
B+C	5	2.99
CRF07-BC	9	5.39
A	3	1.79
CRF52-01B	2	1.20
B+CRF01-AE	7	4.19
CRF01-AE+C	1	5.99
C	1	5.99
CRF67-01B	1	5.99
CRF07-BC	5	2.99
CRF01	1	5.99

**Table 7:** Mutation sites in the protease region and integrase region.

Protease domain	Number of cases (cases)	Integrase domain	Number of cases (cases)
M46N	1	H51Y	1
K43T	1	Y143YC	1
L33LF	1	T97A	1
M184V	1	G140R	1
L33F	3	G118R	1
N88NT	1	S153SF	1
G48R	1	S153SF	1
G73S	1	T197A	2
		E138EK	1
		G140GEKR	1
		G140K	
		G163R	

## Data Availability

The data used to support the findings of this study are available from the corresponding author upon request.
